The article "Antimicrobial potential of two traditional herbometallic drugs against certain pathogenic microbial species" was published in 2016. Journal: BMC Complement Altern Med.

# Antimicrobial potential of two traditional herbometallic drugs against certain pathogenic microbial species

**DOI:** 10.1186/s12906-016-1336-1

**Published:** 2016-09-15

**Authors:** A. U. Wijenayake, C. L. Abayasekara, H. M. T. G. A. Pitawala, B. M. R. Bandara

**Affiliations:** 1 Postgraduate Institute of Science, University of Peradeniya, Peradeniya, Sri Lanka; 2 Department of Botany, Faculty of Science, University of Peradeniya, Peradeniya, Sri Lanka; 3 Department of Geology, Faculty of Science, University of Peradeniya, Peradeniya, Sri Lanka; 4 Department of Chemistry, Faculty of Science, University of Peradeniya, Peradeniya, Sri Lanka

**Keywords:** Rasashastra, Traditional medicine, Antimicrobial, Heavy metals

## Abstract

**Background:**

Mineral based preparations are widely used for centuries as antimicrobial agents. However, the efficacy and the mode of action of mineral based preparations are uncertain due to the insufficient antimicrobial studies. Arogyawardhana Vati (AV) and Manikya Rasa (MR) are such two *Rasashastra* herbo-minerallic drugs commonly in India and other countries in South Asia. Despite of their well known traditional use of skin diseases, reported antimicrobial and mineralogical studies are limited. Therefore, in this study antimicrobial activities of the drugs and their organic, inorganic fractions were evaluated against *Pseudomonas aeruginosa*, *Escherischia coli*, *Staphylococcus aureus*, Methecilline Resistance *Staphylococcus aureus* - MRSA and *Candida albicans*.

**Methods:**

Antimicrobial activity of the drugs, their inorganic residues and organic extracts were determined using four assay techniques *viz* agar well diffusion, modified well diffusion, Miles and Misra viable cell counting and broth turbidity measurements. Mineralogical constituents of the drugs were determined using X-ray diffraction, while total cation constituents and water soluble cation constituents were determined using inductively coupled plasma-mass spectrometer and the atomic absorption spectrophotometer respectively. Thermogravimetric analysis was used to determine the weight percentages of organic and inorganic fraction of the drugs. Particle sizes of the drugs were determined using the particle size analyzer.

**Results:**

AV and MR drugs showed antibacterial activity against both gram positive and gram negative bacterial species when analyzed separately. Inorganic residues of the drugs and organic extracts showed activity at least against two or more bacterial species tested. All tested components were inactive against *C. albicans*. Common mineral constituents of drugs are cinnabar, biotite and Fe-rich phases. Drugs were rich in essential elements such as Na, K, Ca, Mg and Fe and toxic elements such as Zn, Cu and As. However, the water soluble concentrations of the toxic elements were below the detection limits. Both drugs have significantly higher percentages of organic constituents and volatile minerals and particle sizes of drugs are in the nanometer range.

The article "Antimicrobial potential of two traditional herbometallic drugs against certain pathogenic microbial species" was published in 2016. Journal: BMC Complement Altern Med.

**Conclusions:**

AV and MR *Rasashastra* preparations could provide alternatives to synthetic antibiotics against human bacterial infections. Improved solubility and reduced particle sizes are influential physicochemical properties used to enhance the antimicrobial efficacy of the drugs. Therefore, traditional knowledge on the use of antimicrobial mineral sources could provide a novel path for the producing of effective antimicrobial drugs. However, further chemical and toxicological studies are urgently needed for a greater understanding of their toxicity to humans.

## Background

Evolution of microbial resistance, potential health hazards and side effects of exsisting synthetic antimicrobial drugs has led to the investigation of novel antimicrobial agents derived from traditional preparations. Researches in modern medicine have proven that certain metals are effective in antimicrobial functions that cannot be met only by organic molecules [1, 2]. Therefore, mineral based antimicrobial products have recently come into the picture as a potential solution to the rising incidence of drug resistance in microbes [3, 4].

Although some of the metal ions are essential for cellular functions, the same metal ions are toxic to the cells when they are in excess amounts [1]. Certain metal ions bearing natural sources have antimicrobial activity even at very low concentrations and said to have relatively low toxic potential when taken orally [5], these metallic sources have been used as anti microbial agents since ancient times. Sulfides bearing minerals, metal oxides and alumino silicates including biotite mica are some of the minerals that have been used in traditional preparations as metallic antimicrobial sources throughout the world for centuries [6–8].

‘*Rasashstra*’ (Ancient science of alchemy) is the branch of Ayurveda that deals with mineral based drug preparations. In most cases minerals are used as combinations with plant parts, animal by products or any other organic material. Although a few herbometallic traditional preparations possessing antimicrobial activity have been identified, mineral based antimicrobial sources in *Rasashastra* medicine has long been used without much understanding.

Arogyawardhana Vati (AV) and Manikya Rasa (MR) drugs are commonly known herbometallic preparations in the *Rasashastra* medicine, that are prepared by mixing a number of plant parts and purified mineral material [9–12]. AV and MR drugs are traditionally used mainly for skin ailments. In addition, AV is also used to improve appetite and digestion, bowel disorders and as a tonic for heart, liver, uterus, kidneys, intestines [13–18], while, MR is used for allergic conditions, dermatitis, fever, anemia, hiccups and jaundice [13, 19–21].

The article "Antimicrobial potential of two traditional herbometallic drugs against certain pathogenic microbial species" was published in 2016. Journal: BMC Complement Altern Med.

Therefore, these herbo-metallic preparations could have potential to substitute allopathic drugs for the treatment of number of disorders including skin infections caused by microorganism. Hence, the rationalization of specific indications in these products based on their antimicrobial, mineralogical and chemical characteristics is important and useful. Therefore, commercially available AV and MR products were tested for their antimicrobial activities against four bacterial species and one fungal species that are associated with skin diseases, and/or commonly considered as pathogens. Further, the present study was undertaken to investigate the physical and chemical properties of the mineralogical constituents responsible for antibacterial activity.

Among the most common skin pathogens *Pseudomonas aeruginosa* has become known as one of the most problematic gram-negative pathogens with its alarmingly high antibiotic resistance rates [22]. *Staphylococcus aureu*s is another most common human pathogens that leads to many types of infection. This bacterium is responsible for local infections, such as wounds or post operative infection and also for prosthetic infections. *S. aureus* is also known to possess an increasing ability to resist antibiotics such as penicillin, methicillin, tetracycline, erythromycin and vancomycin [23]. *Escherichia coli* are known to be multi resistant bacteria and present in large numbers in the normal intestinal flora of humans, generally causing no harm. However, a number of enteropathogenic strains can cause acute diarrhea, abdominal cramps, nausea and headache. Others have been associated with non-bloody diarrhea, vomiting and fever in infants [22, 24]. Other than the bacterial infections, oral candidiasis and cutaneous candidiasis are common diseases found in the oral cavity and in the folds of the skin caused by fungal infections. Oral candidal infection may spread to the gastrointestinal tract, trachea, lungs, liver and central nervous system opportunistically and capable of causing septicemia, meningitis and endocarditic. Cutaneous candidiasis is found in armpits, hands, groins, buttocks, and under breasts. Among the *Candida* species, *Candida albicans* isolated from oral cavity and skin folds are generally responsible for fungal diseases [2, 25, 26]. Thus, it is necessary and important to evaluation and identify novel alternative herbo-metallic antimicrobial agents for the above causative pathogens for number of ailments including skin and superficial infections.

The article "Antimicrobial potential of two traditional herbometallic drugs against certain pathogenic microbial species" was published in 2016. Journal: BMC Complement Altern Med.

## Methods

### Drug description

“Arogyawardhana Vati” (AV) and “Manikya Rasa” (MR), two *Rasashastra* preparations, were purchased from, Kiriwatthuduwa Liweris Amarathunga company Ltd, a reputed Sri Lankan Ayurvedic preparation center.

### Preparation of extracts

Fractionations of organic and inorganic components of the AV and MR drugs were carried out using a sequential extraction (soxhelt extraction) procedure with hexane (≥99.0 %), dichloromethane (99.6 %) and methanol (≥99.8 %). Extraction period was 24 h for each solvent. All chemicals and solvents used in the experiments were analytical grade high purity solvents from Sigma-Aldrich Company.

### Microbial strains and antimicrobial analysis

All crude extracts, their drugs and residues (inorganic) were used to assess the antimicrobial activity using, agar dilution method, well diffusion assay and a modified version of the same (placing the drug or its components directly on the agar surface), using Mullar Hinton Agar (MHA). The crude extracts were dissolved separately in diluted DMSO (1:7; DMSO: water). Each drug and their components were tested (at 10,000 ppm concentration) against *Pseudomonas aeruginosa* (ATCC-27853), *Escherischia coli* (ATCC 25922)*, Staphylococcus aureus* (ATCC 25923), Methecilline Resistance *Staphylococcus aureus* – MRSA and *Candida albicans* (ATCC 90028), and incubated at 37 °C for 24 h. Inocula of each microbial strain were prepared by suspending 18 to 24 h old cultures in NaCl (0.85 %). Turbidity of each inocular was adjusted similar to 0.5 McFarland standards.

Inocula were flooded onto the surface of Petri plates containing 25 ml of MHA. Wells of 3 mm diameter were cut in the agar using a sterile cork borer. The bases of the wells were sealed by adding a drop of molten agar into each well. Aliquots (100 μl) of the extracts were added into separate wells. Diluted DMSO was used as the negative control. After incubation overnight at 37 °C, the plates were examined and the diameter of the zone of inhibition was measured. A similar test was performed devoid of wells, directly placing and 5 μl suspensions from each extract on the MHA surface as the modified diffusion method.

Inoculated Brain Heart Infusion (BHI) broth cultures of turbidity similar to 0.5 McFarland standard of the above mentioned microorganisms were mixed with the AV and MR drugs (10,000 ppm) and the residues of the drug (remaining solid after the sequential extraction with hexane, dichloromethane and methanol) separately and incubated at 37 °C for 18–24 h in a shaking water bath. The antimicrobial activities of the above components were quantitatively investigated using Miles and Misra method for viability [27] as follows. After incubation 100 μl of the culture was serially diluted and plated on MHA plates. The plates were incubated at 37 °C for 24 h. After incubation, colony forming units (cfu) were recorded in respective dilutions of all the treated samples.

The article "Antimicrobial potential of two traditional herbometallic drugs against certain pathogenic microbial species" was published in 2016. Journal: BMC Complement Altern Med.

The above incubated broth cultures, including the blank samples devoid of drug or residue were centrifuged at 300 rpm for 1 min (sufficient for sediment of the drug or its residue only) and the supernatant (presumably containing microbes) was separated out to test the change in turbidity due to microbial growth by means of absorbance with UV-Visible spectrophotometer. All the experiments were replicated three times. Antimicrobial assays were carried out at the Department of Botany, Faculty of science and Department of Microbiology, Faculty of Medicine, University of Peradeniya, Sri Lanka.

### Mineralogical analysis

Mineralogical compositions of samples were analyzed at the Technical University, Darmstadt, Germany using Siemens D-5000 X-ray Diffraction (XRD) instrument at 40 kV and 34 mA using CuKα radiation of 1.54° A wavelength to determine the properties of crystalline phases of the two drugs. To obtained more precise data with high resolution, samples were analyzed in duplicates with different scanning speeds (1 and 0.1°/min).

Thermogravimetric Analysis (TGA) was performed using Scinco STA N-650 machine to determine the thermal characteristics of the samples. The particle sizes of the drugs were estimated using Marlven Zetasizer nano ZS Particle size analyzer at the Department of Chemistry, University of Peradeniya, Sri Lanka.

### Chemical analysis

Total cation concentration of the two drug samples were determined both by the Inductively Coupled Plasma Mass Spectrometer (ICPMS- Perkin Elmer Sciex ELAN- 6000) and Perkin Elmer-2800 Atomic Absorption Spectrophotometer (AAS) after acid digestion [28] of the inorganic portion of the drugs. The water soluble portion of each drug sample was obtained by filtering each aqueous suspension which was kept in a horizontal shaker at room temperature for 5 h and then allowing equilibrating for 19 h. Analyses of the solutions were carried out on the AAS.

The instruments were calibrated using analytical grade standard solutions of each element. The accuracy of the analytical procedure was evaluated by analyzing reagent blanks routinely with samples as well as by triplication of sub-samples. Detection limits of different elements vary from 1 to 0.001 mg/L for both ICP-MS and AAS. Analyses were done at the Activation Laboratories Ltd. Ontario, Canada and Department of Geology, University of Peradeniya, Sri Lanka, respectively.

The article "Antimicrobial potential of two traditional herbometallic drugs against certain pathogenic microbial species" was published in 2016. Journal: BMC Complement Altern Med.

### SEM analysis

Scanning Electron Microscopic (SEM- EVO - LS15) analysis was carried out in order to determine the bacteria-mineral interactions, morphological changes in microbes and the characteristics of the drugs. Prior to loading the samples for imaging, all the treated samples and untreated bacterial samples (blank) were fixed with formaldehyde for 2 h at room temperature, washed three times with sterilized water and dehydrated twice with an ethanol series, for 10 min at each concentration (30, 50, 70, 80, 90 and 100 %) [29, 30]. To minimize the artifacts during imaging, all bacterial samples were observed under the variable pressure mode. Analyses were done at the Department of Geology, University of Peradeniya, Sri Lanka.

## Results and discussion

### Antimicrobial activity of AV and MR drugs and their organic and inorganic components

In the present study, the in vitro antimicrobial activity of six extracts (hexane, dichloromethane and methanol extracts of two drugs) and four solid components (two drugs and their residues) against five microbial strains, and their antimicrobial activity were qualitatively and quantitatively assessed by the presence or absence of inhibition zones and by the number of colony forming units (cfu). According to the results given in Fig. 1 and Table 1, the extracts of the two drugs investigated showed in vitro antimicrobial activities against some of the bacterial strains tested, explained in detail as follows.

**Fig. 1:** Well diffusion assay against *S. aureus* of (**a**) AV drug, residue and three extracts (**b**) MR drug, residue and three extracts (at 10,000 ppm concentration) H - hexane, Di - dichloromethane, M- methanol, Dr- Drug, Re- inorganic residue of the drug, DMSO- negative control

**Table 1:** Comparison of modified diffusion assay with viable cell count (cfu /ml) of broth cultures incorporated with the drug and residue of AV and MR (10,000 ppm)

Micro organism	Arogyawardhana Vati (AV)									Manikya Rasa (MR)									Control
	Modified diffusion assay					Viable cell count (cfu)				Modified diffusion assay					Viable cell count (cfu)				
	Hexane	Dichloro	Methanol	Drug	Residue	Drug	Residue	LogRcfu		Hexane	Dichloro	Methanol	Drug	Residue	Drug	Residue	LogRcfu		
								Drug	Residue								Drug	Residue	
*P. aeruginosa*	+	+	+	+	+	52 × 10^9^	17 × 10^8^	9	10	vr	vr	+	+	+	5× 10^4^	10 × 10^4^	14	14	10^18^
*E. coli*	+	+	−	+	vr	87 × 10^5^	35 × 10^5^	6	6	+	+	+	+	+	90 × 10^3^	24 × 10^6^	8	5	10^11^
*S. aureus*	+	+	+	+	+	52 × 10^7^	9 × 10^13^	14	8	+	+	+	+	+	63× 10^4^	53 × 10^12^	17	9	10^21^
*MRSA*	+	vr	vr	+	vr	77 × 10^8^	15 × 10^13^	13	8	+	+	+	+	+	26 × 10^4^	33× 10^10^	17	11	10^21^
*C. albicans*	−	−	vr	−	−	15 × 10^6^	14 × 10^6^	0	0	−	−	−	vr	−	4 × 10^5^	45 × 10^7^	1	0	10^6^

*vr* variable results, *+* active, − not active, *LogRcfu* log reduction in colony forming units

The antimicrobial sensitivity of a particular microorganism depended on the type of extract and the type of assay (see Table 1). The hexane extract of AV showed higher antibacterial activity than its dichloromethane and methanol extracts, while the methanol extract of MR exhibited higher antimicrobial activity than the hexane and dichloromethane extracts. Among all tested extracts, the maximum antimicrobial activity was observed with the methanol extract of MR against all the tested strains when considering the clarity of inhibition and the diameter of zone of inhibition. Diluted DMSO, used as the negative control did not show any inhibition zone.

The article "Antimicrobial potential of two traditional herbometallic drugs against certain pathogenic microbial species" was published in 2016. Journal: BMC Complement Altern Med.

None of the extracts or solid components showed antifungal activity against *C. albicans* with the diffusion methods. Nevertheless, a slight reduction (one log reduction) in cfu was noticed in *C. albicans* broth cultures, which were treated with MR drug (Table 1). However, anticandidal activity of a similar drug product named *Hingula manikya rasa* has been reported [9] at 8 mg/ml concentration. This difference may be due to the variable drug preparation techniques and conditions. Further, different particle sizes of the drugs could have an influence on the variable results.

According to the results of Miles and Misra method, highest difference between the control cfu and the corresponding treated broth sample was observed for MR drug against *S. aureus*. Both drugs and residues were active against all the bacterial species when assessed with Miles and Misra method. Antibacterial activity shown by inorganic residues of both drugs with all the tested methods was considerable, indicating that mineral components also have a high influence on antimicrobial activity in addition to the plant extracts.

The broth dilutions were further examined by measuring the turbidity of the microbial cultures using UV-Visible spectrophotometer. The percentage reduction in absorbance (when compared to the control) was compared with the percentage inhibition of the microbial species by Miles and Misra method (viable cell count) (Fig. 2). According to the percentage reduction in absorbance MR drug had the highest antibacterial activity (the greater the values of % reduction, the higher is the activity), while the MR residue showed slightly higher antimicrobial activity than AV residue against *P.aeruginosa*, *S.aureus* and MRSA. Both drugs and their residues did not show significant anticandidal activity. These results tallied with the cfu results obtained by the Miles and Misra method (the grater the value of cfu, the lower is the activity) (Fig. 2). However, in the broth dilution assay the accuracy could be more if the contribution made towards the absorbance values by the non-living microbial cells could be eliminated, from broth culture.

The article "Antimicrobial potential of two traditional herbometallic drugs against certain pathogenic microbial species" was published in 2016. Journal: BMC Complement Altern Med.

**Fig. 2:** Antimicrobial effect of MR and AV drugs and residues by means of cfu and by means of percentage reduction in absorbance at 10,000 ppm concentration level against (**a**) *P. aeruginosa* (**b**) *S. aureus* (**c**) MRSA (**d**) *E. coli* and (**e**) *C. albicans*

### Mineralogical and chemical properties of drug samples

#### Mineralogical properties

XRD analyses show (Fig. 3) that the samples contain characteristically different mineralogical constituents. However, some common minerals such as cinnabar, altered biotite and Fe-rich phases (magnetite, hematite) were recorded from both samples (Table 2). Out of the mineral constituents of drugs, pyrite, magnetite, hematite, altered mica and other sulfide minerals are effective against microbes [31].

**Fig. 3:** X-ray diffraction spectra of (**a**) Arogyawardhana Vati (AV-1, AV-2) and (**b**) Manikya Rasa (MR1, MR2) drugs

**Table 2:** Summary of mineralogical constituents and organic and moisture content of drugs

	AV	Available ions as antimicrobial agents	MR	Available ions as antimicrobial agents
Mineral constituents	Meta cinnabar	S, Hg	Metacinnabar	Hg, S
	Cinnabar	Hg, S	Arsenolite	As
	Arsenolite	As	Sphalerite	Zn, S
	Magnetite/ hematite	Fe	Chalcopyrite/ pyrite	Cu, Fe, S
	Biotite mica (altered)	Fe, Mg, Al, Si	Biotite mica (altered)	Fe, Mg, Al, and Si
Volatile content (wt %)	84 %		70 %	
Moisture content (wt %)	14 %		9.50 %	

Low peak intensities of the XRD patterns indicate that the contents of cinnabar and arsenolite are relatively low in the drugs. A number of metal-alloy and amorphous phases are present (Fig. 3a, b). Since the ingredient minerals used for the preparation of drugs have been subjected to thermal treatments (up to 500 °C), these may be alteration products of some minerals [9, 32]. Due to the inhomoginity of the samples and interferences (with crystalline and amorphos phases) some of the peaks of minerals were hidden during the rapid scanning of the samples. However, the quality of the data was improved and the hidden peaks of some of the minerals were identified by slowing down the scan speed.

Based on the TGA data, the reduction in weight due to the loss of moisture content, organic content and volatile mineral constituents of MR was nearly ~70 % at 450 °C, while the corresponding value for AV drug was 84 % (see Fig. 4).

The article "Antimicrobial potential of two traditional herbometallic drugs against certain pathogenic microbial species" was published in 2016. Journal: BMC Complement Altern Med.

**Fig. 4:** TGA and DSC curves of (**a**) Arogyawardhana Vati (AV) and (**b**) Manikya Rasa (MR) drugs

Although minerals with low boiling points (bp) such as arsenolite (bp; 465 °C) and meta cinnabar (bp; 356 °C) phases could be volatile by the temperature of 450 °C, all the other identified minerals phases are thermally stable in this temperature. Therefore, it could be concluded that a higher fraction of the drugs consist of organic matter while the amount of minerals present in the drugs are relatively lower by weight, despite the antimicrobial activity observed in inorganic residues.

Particle sizes of the MR and AV drugs ranged in between 38–79 and 295–396 nm respectively (Fig. 5). This indicates that both drug particles are small enough to penetrate through the bacterial cell walls.

**Fig. 5:** Percentage number of particle sizes of AV and MR drugs in nanometers

### Major and trace elements

Table 3 represents the cation constituents of the total digested and water soluble portion of AV and MR drugs. Significantly higher concentrations of water soluble Na, K, Ca, Mg and Fe cations were present in both drugs and they can be considered as the available cations contributing to the antimicrobial activity. Although heavy metals such as Zn, Cu and As were present in significant levels in totally acid digested samples, their water soluble concentrations were below the detection limit of the instrument (AAS). In addition, both drugs contained relatively lower amounts of Ag, Mn and Sn metal cations (Table 3) which may contribute towards the antimicrobial activity with the interactions of microbes.

**Table 3:** Cation constituents of totally digested AV and MR drugs and the water soluble portion of AV and MR drugs

Analyte symbol	Total (ppm)		Water soluble (ppm)	
	AV		AV	MR
Mg	5800	4400	1600	3000
K	9100	6300	5600	5000
Ca	13300	3400	3500	1360
Fe	22400	28300	150	110
Na	870	1170	200	500
Al	4800	4100	−	−
Ti	490	340	−	−
S	<1	90000	−	−
P	980	820	−	−
Cu	>10000	>10000	↑	↑
As	12	>10000		
Pb	84.7	351		
Sr	68	25	bd	bd
Zn	169	>10000		
Cd	1.1	1.2		
Cr	53	22	↓	↓
Co	3.5	3.6	−	−
Li	4.4	5.3	−	−
Rb	27.1	24.3	−	−
Mn	237	89	−	−
Sn	85.9	30.6	−	−
Ni	29.2	15.5	−	−
Sb	1.8	160	−	−
Ba	180	7	−	−
Ag	1.5	2	−	−

*bd* below detection limit, − not measured note: data showing the total cation detected from ICP-MS analysis and water-soluble cations detected by AAS

### Probable mechanisms contributory to antimicrobial activity

When considering the antibacterial activities of organic and inorganic constituents of the drugs, it was evident that organic and inorganic components contributed to antimicrobial activity. Therefore, it could be inferred that organic and inorganic components in these *Rasashastra* preparations seem to be synergistically enhancing the antibacterial properties of the drugs.

The article "Antimicrobial potential of two traditional herbometallic drugs against certain pathogenic microbial species" was published in 2016. Journal: BMC Complement Altern Med.

The growth rate of the microorganisms and membrane permeability of the organism to the drug particles can determine antimicrobial activity. Usually fast-growing microbial species are said to have more susceptibility to antibiotics than slow-growing microorganisms [4]. For example, *C. albicans*, a fungus requires more time to proliferate, and hence killing requires additional time than the bacterial species [33]. At the same time drug permeability through the fungal membranes are much slower than the bacterial membranes. This could be an explanation for the poor or no activity noticed against *C. albicans* with the tested components, in the current study.

### Assay type based antimicrobial activity- contradictions and suggestions

Evan though, the diameter of zone of inhibition in the well diffusion assay and clarity of the zones in modified diffusion assay were used to evaluate the antimicrobial activity of the plant extracts with inorganic residues and drugs (inorganic and organic components as a mixture), it should be noted that the diffusion abilities are different in components. As the different components have different abilities to diffuse through the selected medium these differences may contribute to the strength of antimicrobial action of a particular extract. However in this study, particular assays have been done only to determine the contribution of each component (extracts, drugs and residues) towards the antimicrobial activity.

In discussing the assays based on partially soluble solid materials, it is recorded that broth dilution method is the best method to estimate the approximate potency of a particular compound within a given period of time under given pH values [34]. Therefore, the methodology employed needs to be considered in more depth in antimicrobial assays. From this point of view, further investigations are required to improve the antimicrobial methods for the partially soluble solid components and plant extracts.

### Physiochemical characteristics of the drugs

Several important physiochemical properties of the mineral constituents of AV and MR drugs were observed that could influence antibacterial activity viz particle sizes, different shapes of particles which are favorable for antimicrobial activity (Fig. 6a, b), exchangeable and soluble elements and the mineral phases (oxides, sulfides, silicates, metal alloys) of the inorganic constituents.

**Fig. 6:** SEM images of (**a**) AV drug rich in rounded shaped aggregates of nano-size particles and randomly distributed elongated grains of minerals (**b**) MR drug consisting of aggregates of acicular, triangular, rounded and irregular shaped nano-size particles rich in metal sulfides

Physical interaction with the microbial cell surface is a most striking factor that contributes to the antimicrobial activity of a particular particle. Small particles sizes have a major influence against antimicrobial activity. Importance of particle size of the drugs is evident when the antibacterial activity of the drugs is compared with their particle sizes. Both MR and AV drugs consisted of fine particles. Further, MR drug with relatively smaller particles showed higher antibacterial activity than AV drug with slightly larger particles. It has been observed that antimicrobial activity increased with the decreasing particle size by many previous studies on metallic antibiotics [35, 36]. Previous studies suggested that the enhanced antimicrobial activity is due to the ease of interaction and penetration of small particles (sizes ranging from 10 to 80 nm) into bacterial membranes [23]. Other than the particle size their shapes and surface charge that control the release of metal ions from the drugs, play a role in microbial toxicity [1]. Importances of the shapes of nano drug particles as antimicrobial agents have been shown by Pal et al., [37]. It is recorded that the highly reactive triangular shaped nano-particles with antimicrobial activity compared to the rounded and rod shaped particles. They have explained the differences in the observed trends in inhibition with the shapes in terms of the percent active faces present in nano-particles with different shapes. Therefore, considering the shapes of AV and MR drug particles, MR drug could be more reactive than AV as MR consisted of differently shaped particles in comparison to AV (Fig. 6a, b). In addition, as observed in the current research, all bacterial species showed inhibition zones with AV and MR residues, when directly placed over the microorganisms in the modified diffusion assay. It could be suggested that antibacterial action of inorganic residues may have been induced due to the effective physical nature of the processed mineral particles.

The article "Antimicrobial potential of two traditional herbometallic drugs against certain pathogenic microbial species" was published in 2016. Journal: BMC Complement Altern Med.

In addition to inheritent antimicrobial properties of inorganic residues, the organic constituents may have promoted the antimicrobial action of mineral constituents by increasing the release of the antimicrobial metal cations in to the growth medium. Since, most of the antimicrobial plant constituents possess slightly acidic pH values (around pH 5), the releasing capacity of metalic constituents could be enhance by the organic matter in drug mixtures. Further, acidic medium provided by the organic constituents could enhance the cell membrane permeability of the bacteria [38]. Therefore, metallic constituents can easily reach the targeted bacterial sites. In addition to the action of pH, plant constituents could contribute to the number of antibacterial mechanisms leading to microbial lethality. However, the action of organic constituents of the drugs cannot be elaborated here due to the complexity of the combinations of organic matter.

### Evaluating antibacterial process / possible mechanisms

Significant alterations in treated bacterial samples were observed by SEM. The electron micrographs of treated bacteria (*S. aureus* and *E. coli*) samples are shown in Fig. 7. In a view of Fig. 7b shrinked cells of *S. aureus* can be seen attached to the surface of AV drug particles, *S. aureus* treated with MR drug showed (Fig. 7c) relatively higher damage to cells compared to the AV treated *S.aureus*. Similarly, MR treated *E.coli* (Fig. 7f) showed a stronger growth inhibition compared to the AV treated *E.coli* (Fig. 7e). These SEM observations tally with the results obtained from the antimicrobial assays which showed higher inhibition effect of MR drug compared to the AV drug. Altered microbes with both drugs had either relatively flattened and elongated or shorter and more compact shapes compared to their untreated bacterial controls (Fig. 7a and d). F). Shortening of the bacterial cells (Fig. 7b) indicates that treated bacteria was not able to grow to maximum length; whereas expansion and elongation of the cells (Fig. 7e) could be a result of accumulation of drug particles inside the cell wall or extra hydration of the bacterial cells.

**Fig. 7:** SEM images of (**a**) cocci shaped cells of untreated *S. aureus* with smooth, intact surfaces. **b** altered *S. aureus* cells after treating with AVdrug (**c**) highly altered *S. aureus* cells after treating with MR drug (**d**) bacilli shaped cells of untreated *E. coli* (**e**) altered *E. coli* with cracked and damaged bacterial cell wall after treating with AV drug (**f**) completely destroyed *E. coli* cells after treating with MR drug

Antibacterial activity of AV and MR could be directly related to the actions of their metal oxide, pyrite, mica, cinnabar and other sulfide mineral phases. Although antimicrobial mechanism should be considered in combination, possible effect of most influential minerals are discussed individually based on literature (Table 4).

**Table 4:** Possible antimicrobial mechanisms of minerals in MR and AV drugs

Mineral	Mechanism of action
Pyrite/ chalcopyrite	Spontaneously generate hydrogen peroxide (H_2_O_2_) and hydroxyl radicals when they are placed in water. Caused to degrade ribosomal RNA and DNA [45].
Sulfur present in soluble forms with water	Could interact with the oxygen radicals in the drug-microbe aqueous mixture which may in turn be transformed into pentathionic acid (H_2_S_5_O_6_), which could be a source of the antibacterial activity of water based broth preparations [46, 47].
Oxides (zinc, copper and iron oxides)	Could act as sources that create hydrogen peroxide oxide radicals which contribute to the inhibition of both gram positive and negative bacterial species [48].

In addition to the contribution of the well-known antibacterial constituents described in Table. 4, processed mica (Abhrak bhasma) individually possesses antibacterial activity against *S. aureus* and MRSA in the aqueous medium [39]. Therefore, the water soluble cations in mica might have contributed to the antibacterial activity rather than its solid constituents [40, 41]. Further, surface charges of minerals can interact with bacteria [42, 43]. Bacteria (negatively charged) can be easily attracted to the mineral surfaces with positive charges by the electrostatic interaction. Therefore, minerals present in the oxidized form in the drugs (iron oxides and other metal oxides) could contribute to damage the bacterial cell wall and increases permeability to other materials.

The article "Antimicrobial potential of two traditional herbometallic drugs against certain pathogenic microbial species" was published in 2016. Journal: BMC Complement Altern Med.

Overall, it can be suggested that the growth inhibition and cellular death of microorganisms are a result of a combination of different mechanisms. Further, depending on the chemistry of the minerals/metals, the mechanisms of antimicrobial activity may differ in the two drugs assessed.

### Effect of toxic metals

Metal concentrations were determined only for the inorganic residues in the current study. For 1 g of each drug, the mineral constituents were <0.16 and <0.3 g for AV and MR respectively. Therefore the oral dosage of these drugs used in the current study could have lower metal toxicity than the observed values with cation analysis. Kumar et al.*,* [13], have carried out safety evaluation of Arogyavardhini vati (AV) on brain, liver and kidney in rats using different oral doses of 50, 250 and 500 mg/kg (one, five and ten times of human equivalent dose respectively) and there results have revealed that AV in the doses equivalent up to ten times of the human dose administered to rats for 28 days does not have appreciable toxicological effects on brain, liver and kidney. Further their studies on safety of AV (500 mg) treatment [44] for dyslipidemia patients (87) by assessing hepatic function (aminotransferase [ALT], aspartate transaminase [AST], alkaline phosphatase [ALP], bilirubin, and β^2^ microglobulin), renal function (urea and creatinine and NGAL) tests, and urine mercury level have shown that there is no significant change in serum ALT, AST, ALP and bilirubin, urea, creatinine β^2^ microglobulin, and NGAL levels at the end of study as compared to the baseline levels. Therefore, they have concluded that AV treatment is safe and effective for dyslipidemia.

The article "Antimicrobial potential of two traditional herbometallic drugs against certain pathogenic microbial species" was published in 2016. Journal: BMC Complement Altern Med.

In addition, previous investigations carried out on the genotoxic potential of Manikya Rasa (MR) (2000 mg/kg), in Wistar rats by Micronucleus assay and Comet assay revealed the lack of induction of micronuclei or DNA damage despite the presence of traces of transformed toxic heavy metals in these formulations [45, 46].

Although, there are many supportive studies recorded on the minimal cytotoxicity of the AV and MR drugs it is necessary to remove or replace the toxic cations in the drugs such as Cu, As, Zn, Pb, Sn and Hg (Table 4) by antibacterial cations which are free of adverse effects in the oral applications. In addition, toxicity of the drugs can be minimized by reducing the effective dose of the drugs with the improvement of the pharmaceutical qualities such as high specific surface area (by increasing the fine fraction of the particles) and solubility. Further, care should be taken to select the raw materials with minimal toxic substances. Oral use of these drugs without the knowledge of their composition could be harmful [5]. Therefore, these drugs should be tested for the threshold values of cationic constituents prior to the applications.

## Conclusions

AV and MR drugs have antibacterial potential against tested gram positive (*Staphylococcus aureus* and MRSA) and gram negative (*Pseudomonas aeruginosa*, *Escherichia coli*) bacterial species. Our analyses suggest that mineral and herbal constituents in the AV and MR *Rasashastra* drugs contribute to the antibacterial activity. Therefore, AV and MR *Rasashastra* preparations could provide alternative treatments to synthetic antibiotics against human bacterial infections. AV and MR drugs possess a number of physical and chemical characteristics, such as small particle sizes and higher water solubility which contribute to enhance the antimicrobial mechanisms.

Even though these traditional herbo-metallic preparations seem to hold great promise for their antimicrobial efficacy, further biochemical and toxicological studies are needed for a greater understanding of their toxicity to humans.

## Abbreviations

AAS: Atomic absorption spectrophotometer
ATCC: American type culture collection
AV: Arogyawardhana Vati
BHI: Brain heart infusion
cfu: Colony forming unit
ICPMS: Inductively coupled plasma mass-spectrometer
MR: Manikya Rasa
MRSA: Methecilline resistance *Staphylococcus aureus*
TGA: Thermal gravimeter
XRD: X-ray diffractrometer

The article "Antimicrobial potential of two traditional herbometallic drugs against certain pathogenic microbial species" was published in 2016. Journal: BMC Complement Altern Med.

## References

[1] Lemire JA, Harrison JJ, Turner RJ (2013). Antimicrobial activity of metals: mechanisms, molecular targets and applications. Nat Rev Microbiol.

[2] Anuphrab SS, Srikhiran T, Thaweboon B, Thaweboon S, Amomasakchai T, Dechkunakorn S, Suddhasthira T (2013). Antimicrobialeeffects of silver zeolite, silver zirconium phosphate silicate and zirconium phosphate aginest oral microganisams. Asian Pac J Trop Biomed.

[3] Azam A, Ahmed AS, Oves M, Khan MS, Habib SS, Memic A (2012). Antimicrobial activity of metal oxide nanoparticles against Gram-positive and Gram-negative bacteria: a comparative study. Int J Nanomedicine.

[4] Hajipour MJ, Ashkarran AA, Aberasturi DJ, Lrramendi IR, Serpooshan V, Parak WJ, Mahmoudi Mand Rojo T (2012). Antibacterial properties of nanoparticles. Trends Biotechnol.

[5] Liu J, Shi JZ, Yu LM, Goyer RA, Waalkes MP (2008). Mercury in traditional medicines: is cinnabar oxicologically similar to common mercurials?. Exp Biol Med (Maywood).

[6] Zhou X, Zeng K, Wang Q, Yang X, Wang K (2010). In vitro studies on dissolved substance of cinnabar: chemical species and biological properties. J Ethnopharmacol.

[7] Miao JW, Liang SX, Wu Q, Liu J (2011). Toxicological evaluatin of realgar containing Niu-Huang-Jie-Du Pian as compared to arsenicals in cell cultures and in mice. ISRN Toxicol.

[8] Wu J, Shao Y, Liu J, Chen G, Ho PC (2011). The medicinal use of realgar (As_4_S_4_) and its recent development as an anticancer agent. J Ethnopharmacol.

[9] Prabhakar IM, Ranjan PR (2013). Preperation and phisicochemical characterisation of hingula manikya rasa. Int J Res Ayurveda Pharm.

[10] Bhattacharya B (2011). Elucidating the nanomaterialistic basis for Ayurvedic Bhasmas using physicochemical experimentation. J Biomed Nanotechnol.

[11] Rajput D (2013). Ayurvedic view on heavy metal poisoning with special reference to Naga bhasma incinerated lead, a literary study. Int J Pharm Biol Arch.

[12] Sharma R, Amin H, Ruknuddin G, Prajapati PK (2015). Efficacy of Ayurvedic remedies in type 2 diabetes: a review through works done at Gujarat Ayurved University, Jamnagar. J Med Nutr Nutraceut.

[13] Kumar G, Srivastava A, Sharma SK, Gupta YK (2012). Safety evaluation of an Ayurvedic medicine, Arogyavardhini vati on brain, liver and kidney in rats. J Ethnopharmacol.

[14] Rao GP (2008). A text book of Bhaisjya Kalpana Vijnanam.

[15] Dwivedi ML, Tripathi SV, Dwivedi HS (1984). Role of Phaltrikadi kashaya and arogyavardhini vati in the treatment of jaundice (Kamala). Sachitra Ayurved.

The article "Antimicrobial potential of two traditional herbometallic drugs against certain pathogenic microbial species" was published in 2016. Journal: BMC Complement Altern Med.

[16] Wada O, Yamaguchi N, Ono T, Nagahashi M, Morimura T (1976). Inhibitory effect of mercury on kidney glutathione peroxidase and its prevention by selenium. Environ Res.

[17] Sarashetti DR, Ahmed DIS (2010). Physico chemical analysis and evaluation of antibacterial and anti fungal activity of Arogyavardhini Vati RGUHS.

[18] Hegde P, Hemanth D, Emmi S, Shilpa M, Shindhe P, Santosh Y (2010). A case discussion on eczema. Int J Ayurveda Res.

[19] Kumar G, Srivastava A, Sharma SK, Gupta YK (2014). The hypolipidemic activity of Ayurvedic medicine, Arogyavardhini vati in Triton WR-1339-induced hyperlipidemic rats: a comparison with fenofibrate. Indian J Med Res.

[20] Inamdar MP, Patil RR, Mhaske RH, Singh SRP (2013). Study of antifungal activity of hinguliya manikyarasa in *Candida albicans* by its various concentrations. Int J Res Ayurveda Pharm.

[21] Sud S, Sud KS (2012). Acute and sub-acute toxicological study of rasa manikya prepared with classical-modified and adopted method. Anc Sci Life.

[22] Tekwu EM, Pieme AC, Beng VP (2012). Investigations of antimicrobial activity of some Cameroonian medicinal plant extracts against bacteria and yeast with gastrointestinal relevance. J Ethnopharmacol.

[23] Tran NO, Mir D, Sinha A, Nayar S, Webster T (2010). Bactericidal effect of iron oxide nanoparticles on *Staphylococcus aureus*. Int J Nanomedicine.

[24] Nataro JP, Kaper JB (1998). Diarrheagenic Escherichia coli. Clin Microbiol Rev.

[25] Méan M, Marchetti O, Calandra T (2008). Bench-to-bedside review: Candida infections in the intensive care unit. Crit Care.

[26] Vincent JL, Anaissie E, Bruining H, Demajo W, el-Ebiary M, Haber J, Hiramatsu Y, Nitenberg G, Nyström PO, Pittet D, Rogers T, Sandven P, Sganga G, Schaller MD, Solomkin J (1998). Epidemiology, diagnosis and treatment of systemic Candida infection in surgical patients under intensive care. Intensive Care Med.

[27] George AT, Namasivayam SK, Raju S (2013). Synthesis, characterization and anti bacterial activity of chitosan stabilized nano zero valant iron. BOPAMS.

[28] Blacerzak M (2002). Sample digestion methods for determination of traces of precious metals by spectrometric techniques. Anal Sci.

[29] Milani M, Drobne D, Tatti F, Vilas M, Díaz J (2007). How to study biological samples by FIB/SEM?.

[30] Fratesi SE, Lynch FL, Kirkland BL, Brown LR (2004). Effects of SEM preparation techniques on the appearance of bacteria and biofilms in the Carter Sandstone. J Sediment Res.

[31] Metge DW, Williams L, Eberl DD, Bium AE, Harvey BW. Synthetic antibacterial clay compositions and method of using same. United States Patent US 2013/0004544 A1. 2013.

[32] Yang LH, Hong ZS (2005). Detection of mineralogical changes in pyrite using measurements of temperature-dependence susceptibilities. CHJG.

The article "Antimicrobial potential of two traditional herbometallic drugs against certain pathogenic microbial species" was published in 2016. Journal: BMC Complement Altern Med.

[33] Baillie GS, Douglas LJ (1998). Effect of growth rate on resistance of *Candida albicans* biofilms to antifungal agents. Antimicrob Agents Chemother.

[34] Rios JLR, Recio MC (2005). Medicinal plants and antimicrobial activity. J Ethnopharmacol.

[35] Khurana C, Vala A, Andhariya N, Pandey OPCB (2014). Antibacterial activity of silver: the role of hydrodynamic particle size at nanoscale. J Biomed Mater Res A.

[36] Uskokovic V, Batarni SS, Schweicher J, King A, Desai TA (2013). Effect of calcium phosphate particle shape and size on their antibacterial and osteogenic activity in the delivery of antibiotics in vitro. Appl Mater Interfaces.

[37] Pal S, Tak YK, Song JM (2007). Does the antibacteria lactivity of silver nanoparticles depend on the shape of the nanoparticle? A study of the Gram-negative bacterium Escherichia coli. Appl Environ Microbiol.

[38] Gyawali R, Ibrahim SA (2014). Natural products as antimicrobial agents. Food Control.

[39] Wijenayake AU, Pitawala HA, Bandara BR and Abayasekara CL. Antimicrobial activity and chemical and mineralogical characters of a mica based herbo-metallic drug. Sri Lanka: Peradeniya University Research Sessions (iPURSE); 2014.

[40] Otto CC, Haydel SE (2013). Exchangeable ions are responsible for the in vitro antibacterial properties of natural clay mixtures. PloS One.

[41] Williams LB, Metge DW, Eberl DD, Harvey RW, Turner AG, Prapaipong P, Poret-Peterson AT (2011). What makes a natural clay antibacterial?. Environ Sci Technol.

[42] Lower SK, Tadanier CJ, Hochella MF (2001). Dynamics of the mineral–microbe interface: use of biological force microscopy in biogeochemistryand geomicrobiology. Geomicrobiol J.

[43] Guo T, Cao S, Su RS, Li Z, Hu P, Xu Z (2011). Adsorptive property of Cu2+loaded montmorillonite clays for Escherichia coli K88 in vitro. J Environ Sci.

[44] Kumar G, Srivastava A, Sharma SK, Gupta YK (2016). Safety and efficacy evaluation of Ayurvedic treatment (Arjunapowder and Arogyavardhini Vati) in dyslipidemia patients: a pilot prospective cohort clinical study. AYU.

[45] Sathya T, Murthy B, Vardhini N (2008). Genotoxicity evaluation of certain Bhasmas using micronucleus and Comet assays. Internet J Altern Med.

[46] Vardhini NV, Sathya TN, Murthy PB (2010). Assessment of genotoxic potential of herbomineral preparations-bhasmas. Curr Sci.

[47] Cohn CA, Laffers R, Simon SR, Riordan TO, Schoonen MA (2006). Role of pyrite in formation of hydroxyl radicals in coal: possible implications for human health. Part Fibre Toxicol.

[48] Gheresetich I, Benedetta MD, Hercogova MJ, Lotti TM (2001). Mineral waters: instead of cosmetics or better than cosmetics?. Clin Dermatol.

